# Nexus Between Consumer’s Motivations and Online Purchase Intentions of Fashion Products: A Perspective of Social Media Marketing

**DOI:** 10.3389/fpsyg.2022.892135

**Published:** 2022-06-22

**Authors:** Feng Yu, Qian Wenhao, Zhou Jinghong

**Affiliations:** School of Public Economics and Administration, Shanghai University of Finance and Economics, Shanghai, China

**Keywords:** young consumers, consumer motivations, commitment, fashion products, social media

## Abstract

This study aimed to investigate the effects of customers’ motivations (specifically young consumers) on online purchase intentions as mediated by commitment toward online fashion retailers. The survey method was used to collect data from Chinese respondents using a questionnaire. The convenience sampling technique was used to collect data from 275 respondents. Collected data were analyzed on smart-PLS using the structural equation modeling technique. Results of the study show a significant and positive impact of social empowerment and remuneration motivations on consumer commitment online purchase intention. Further results show that consumer commitment partially mediates the relationship between social empowerment, remuneration, and online purchase intention. This study contributes to the literature in the domain of consumer commitment by focusing on the underlying needs and motivations of consumers. The researchers have demonstrated a strong need to understand the dynamics of commitment due to its importance in affecting purchase intention. This study also has several implications that guide online retailers how to motivate consumers with social, remuneration and empowerment incentives to develop their intention to purchase online. Fashion retailers are suggested to gratify certain consumer motives to increase commitment. Specifically, among the three motives, empowerment motivation emerged as the strongest predictor of consumer commitment in social media environment. This study will help to the online brands to attract more customers by providing the motivation such financial, empowerment and socialization.

## Introduction

Social media has become an important and influential means of communication in our current age, with millions of people and organizations using it. While many academicians and practitioners in marketing are interested in this new form of communication, they actively research and uncover the unique issues and advantages that come with it (Li et al., 2021b). For example, customers are currently purchasing in different ways, finding online. In addition to that, they are also visiting physical locations to compare products and prices, using smartphones and tablets, webpages to locate their best choices, and using various devices to help them find the most beneficial purchase (Haque and Mazumder, 2020). As communication channels have expanded, companies have needed to maintain adequate customer service in a digital world that become more challenging, so research has become a necessity to help firms meet this demand (Jamil et al., 2021a). To keep up with consumer behavior that is so fluid, it is essential to consider better the antecedents or variables influencing customer purchasing intention. Even if the Internet makes it easy to gather and present vast amounts of information, but, in today’s busy, chaotic shopping world, it is not easy to catch customers’ interest and have an impact on their purchasing decisions (Cao et al., 2021).

While companies and customers both demand and desire greater convenience in shopping, making the purchase process more complicated, customers also want to use the Internet as a primary source for purchasing (Gautam and Sharma, 2017; Jamil et al., 2021). While buying patterns on the Internet have been mentioned previously, the similarities and differences between Internet buyers have not been adequately studied. As it is thought that customers need more adaptability and have complete access to the merchandise is considered to be a significant factor on why people choose to purchase online, so greater convenience and improved choice are the main drivers to purchase online (Chen and Lin, 2019). However, researchers and professionals study online consumers’ attitudes and actions and cover various aspects, ranging from the conflicting outcomes of research to online consumer motives, such as remuneration, social and empowerment motivations leading to consumer commitment (McClure and Seock, 2020).

This study is particularly commenced to check the consumer’s motivations behind their intention to purchase online. Psychological motivation and marketing are the main areas of study that target consumer behavior. Several scholars defined motivation, but the closest definition of motivation that best suits our research is motivated to achieve goals. Therefore, understanding the consumer’s motivation behind online retailing is a crucial subject to study. Previously conducted studies confined consumer’s motivation in their general online activities. However, from a business perspective, there is a lack of literature on consumer motivation. On the basis of above explanation, we draw the following questions which need to be discussed in this study:

*RQ1:* What is the impact of consumer motivations on purchase intention is social media settings?

*RQ2:* How consumer commitment mediates the relationship between consumer motivations and purchase intention in social media setting?

Furthermore, prior studies mainly concerned the impacts of utilitarian and hedonic motivations on consumers’ engagement in online and social media settings. If we specifically talk about social media marketing campaigns, remuneration and social motivation concepts are still not thoroughly studied. Last but not least, the researcher also identified little empirical evidence of empowerment motivation in social media-mediated marketing environments (Irshad et al., 2020). Therefore, this research aims to examine the impact three consumer motivations (i.e., social, empowerment, remuneration) on social media and the online purchase intentions of customers to increase their commitment toward retailers/brands. Furthermore, the study also aims to evaluate the mediating effects of consumer commitment on consumer motivation and online purchase intentions.

Using the uses and gratification (UGT) theory and theory of reasoned action (TRA) this study focused on consumers motivation and its impact on purchase intention of fashion products in social media settings. Targeted population of this study was the university students and those universities are in metropolitan city Shanghai. This study finds that there is positive and significant relationship between consumer motivations and purchase intention as well as customer commitment mediates between consumer motivation and purchase intention of fashion products.

The following paragraphs review relevant literature and are followed up by the hypothesized relationships between constructs. Then the research methods, analyses, and findings are recorded and discussed. Finally, both the theoretical and managerial implications and the limitations and directions for future research have been discussed.

## Literature Review

### Theoretical Background

Social media marketing uses social media networks to produce, communicate, supply, and share products of interest to a company’s stakeholders. Social media marketing consists of some motive components from applications and awards (Perugini and Solano, 2021). Uses and Gratification Theory (UGT) is one of the most popular theories to explain consumer desires and the effects of different behavioral intentions. The main objective of UGT is to demonstrate why diverse desires and motivations prompt people to use a medium to meet these needs (Khoa, 2020). UGT applicability in social media marketing is strongly promoted by scholars to consider customer desires (Santos Corrada et al., 2020). Past research has examined the correlation between UGT and consumers’ motives (utilitarian and hedonic) to investigate the connection between motivation and various behavioral effects, such as whether or not consumers would go on brand pages and the interaction with social media material with regard to like, posting and sharing (Hossain et al., 2019). We, therefore, consider the UGT to be a suitable structure to analyze the effect on online buying intentions of user motives (i.e., social, remuneration and empowerment). In this study, we are also gathering insights into our research model based on the theory of reasoned action (TRA). The TRA states that the intention of customers to conduct themselves is impaired by conduct as a commitment (Ibrahim, 2021). Researchers evaluated the TRA empirically by extracting TRA elements such as commitment and purchasing intentions in the web and social media setting. According to Zhao et al. (2019), the TRA may be used in studies examining commitment, as commitment can be perceived as a preceding belief factor affecting an individual’s online purchase intentions. Similarly, other researchers have used the TRA as a computational tool to empirically examine the association between commitment and purchasing intentions in a social media context (Yee et al., 2021). Thus, we use UGT and the TRA to demonstrate how antecedents such as motivations and commitment can significantly impact consumers’ online purchase intentions in a social media context (Wu and Kuang, 2021).

### Hypotheses Development

#### Remuneration Motivation, Customer Commitment, and Online Purchase Intention

The desire to get rewards through promotional deals, free coupons, and other loyalty incentives contribute to remuneration motivation. Promotional incentives are considered essential predictors of consumer responses to any marketing offer and contribute to positive purchasing intentions (Femenia-Serra and Gretzel, 2020; Jamil et al., 2021b). The consumer commitment to retailers/brands has been very beneficial in the ordinary sense of providing customer benefits in online settings. McClure and Seock (2020) found commitment a positive psychological association with a retailer/brand. Three aspects of commitment, normative, affective, and continuous, are presented in organization commitment theory. Affective commitment is an emotional relationship that leads a customer to a specific behavior (Muralidharan and Men, 2015; Gul et al., 2021a). This transfer could be a repeated purchasing activity, and I would prefer to shop online in the context of social media. Rather (2019) noted that commitment could be described as a wish of the member to continue its relationship with the retailer/brand through the online purchases. Cao et al. (2021) illustrate commitment as a ‘practical part of the social identity of online purchase. Wei et al. (2016) emphasized the need for an empirical study of the impact of remuneration motivations on commitment and online purchase intentions in social media marketing (Mustafa et al., 2022a). We suggest that if retailers/brands in social media meet the remunerative needs of consumers, they can continue to build a commitment and even encourage the buying intentions of customers online. Therefore, it is hypothesized that:

*H1a:* Remuneration Motivation has a positive impact on consumer commitment toward online purchasing.

*H1b:* Remuneration Motivation has a positive impact on the online purchase intention of consumers.

#### Social Motivation, Customer Commitment, and Online Purchase Intention

In various usage situations, peer influence occurs. Peers impact customers’ ethical and monetary behaviors (Bazi et al., 2020). Young consumers also visit digital media in Asia-Pacific to follow their peers’ views to test the credibility of online content. As social networks develop, interactions and partnerships have come true with like-minded peers, and now people can exchange or search for product knowledge from social networks and even strangers (Yang and Che, 2020). People can share their experiences and thoughts on social media goods, and modeling can occur where the customer accepts the advice of their peers for acceptance (Wang et al., 2015). However, the effect of peer contact on obligations and the online buying intentions of consumers through social media has barely been investigated. We expect customer input from peers on social media retailers/brands to help shape their commitment and improve online shopping intentions. Therefore, it is hypothesized that:

*H2a:* Social Motivation has a positive impact on consumer commitment toward online purchasing.

*H2b:* Social Motivation has a positive impact on the online purchase intention of consumers.

#### Empowerment Motivation, Customer Commitment, and Online Purchase Intention

Empowerment refers to the need for the position of the opinion maker to influence other customers or products (Tajurahim et al., 2020; Awan et al., 2021a). Social networking is an effective way of expressing customer views and calling for brand improvements. Empowerment has been noticed as a catalyst in brand SNS pages. While the topic of empowerment in social sciences has been widely discussed, the empowerment of consumers has not yet primarily been explored in a consumer environment (Naiwen et al., 2021; Li et al., 2021a). The impetus for empowerment is focused on persons who use online media to influence or exert control over others. Lin et al. (2019) discussed that although the well-informed buyers of the present time cannot just be perceived as the marketers’ target, their effect on marketing activities often warrants close attention. The explosion of emerging Internet technology has allowed users to gain greater insight and freedom of choice than ever before (Awan et al., 2021b).

Consumer empowerment can be described as feeling ‘voluntary in actions,’ to support one’s behavior entirely and authentically, and to be the originator of one’s conduct. This description means that the client feels independence without the psychological pressure and considers his or her behavior (Buzeta et al., 2020; Gul et al., 2021b). Autonomy can be mirrored in customer behavior in the sensation of empowerment to influence a behavior’s results. Social media play a crucial role in enabling consumers to broaden their voices worldwide (Mustafa et al., 2022b). Companies may use empowerment approaches to gather ideas, responses, and input from customers on innovation in products and processes. According to Mostafa (2021), empowering the modern age will contribute to significant goals, attitudes, and behavioral benefits. The participation of social media of a vast number of different retailers has resulted in greater competition (Naseem et al., 2021). Thus, to maximize customer commitment and online purchasing intentions, it has become essential for retailers to accept user feedback regarding their products and services. Therefore, it is hypothesized that:

*H3a:* Empowerment Motivation has a positive impact on consumer commitment toward online purchasing.

*H3b:* Empowerment Motivation has a positive impact on the online purchase intention of consumers.

#### Consumer Commitment and Online Purchase Intention

As marketers are trying to develop consumer strategy and establish partnerships over time, consumers may deviate from brand commitments with little or no switching costs due to the ready availability of affordable branded products. Therefore, one of the company’s ultimate aims is to resolve this discrepancy and effectively fulfill the brand promise in the new, highly competitive, and diverse marketplace (Morgan and Hunt, 1994). Recently, researchers have said that market management transforming brand experience into customer commitment is one of the most critical issues. Commitment is an essential function and a condition for achieving a company’s goals. Without a solid commitment base, a healthy customer partnership cannot effectively be established. The Consumers’ commitment applies to the willingness of the consumer to continue their association with the retailer/brand (Rehman et al., 2019; Gul et al., 2021c).

Commitment is critical in online purchases because many users in social networks also give their views on various retailers’ goods and services (Chetioui et al., 2021; Mohsin et al., 2021b). Therefore, it can be assumed that purchases that are conducted *via* social media often entail a consumer’s commitment in retailers operating in social networks to complete effective transactions, much as any other online business where commitment is the critical determinant of purchase intentions (Oghazi et al., 2018; Awan et al., 2021c). Therefore, we believe that there is significant value to commitment in social media environments, which will make customers think about purchasing the product. Consequently, it is hypothesized that:

*H4:* Consumer Commitment has a positive impact on consumer’s purchase intention.

#### The Mediating Role of Customer Commitment

Morgan and Hunt (1994) propose that commitment requires vulnerability, and therefore parties are encouraged to find trusted partners. Show that confidence in their service providers has a significant commitment to the relationship between customers. Rehman et al. (2019) also argues that trust is one of the most critical determinants of commitment to ties. There is well established in the marketing literature the constructive association between relationship constructs (i.e., commitment) and desirable actions. Show that the buying company’s interest in the supply company is positively linked to a potential relationship with the buying company. The Commitment was seen to be positively related to good motives such as repeated purchases, recommending, insensitive pricing actions, and cross-buying (Wei et al., 2016; Mohsin and Ivascu, 2022).

However, there is also a great deal of unexplored debate about customer commitment to retailers in social media as a basis for influencing the relationship between consumer motivations and their online purchasing intentions. Commitment is crucial in alleviating uncertain emotions, as it is a vital driving force for online buying by consumers (Shujaat et al., 2021). When their needs are satisfied, consumers will cultivate good behavioral intentions (e.g., purchasing intentions). However, if the commitment feature is lacking, users would be less receptive to online purchases (Rehman et al., 2019). This study hypothesized that the relationship between customer motivations and intentions to purchase online is mediated by commitment to social media retailers. Therefore, it is hypothesized that:

*H5a,b,c:* Consumer commitment mediates the relationship between (a) remuneration motivation, (b) social motivation, (c) empowerment motivation, and online purchase intention of consumers (Figure 1).

**Figure 1:** Conceptual framework.

## Research Methodology

A self-administered questionnaire was used to collect data from respondents. A pilot study with 30 participants was carried out. Since providing recommendations, revisions were made to the final questionnaire to make it more understandable for the study’s respondents. To ensure the content validity of the measures, three academic experts of marketing analyzed and make improvements in the items of constructs. The experts searched for spelling errors, grammatical errors and ensured that the things were correct. The experts have proposed minor text revisions to social motivation and consumer commitment items and advised that the original number of items be maintained. Researchers took the services of a Chinese language expert as volunteer to translate the questionnaire in Chinese language too. Questionnaire is divided into two columns one is in English language and second is in Chinese language for the understanding of Chinese respondents. Convenience sampling technique was employed to select the study participants because a list of all buyers of fashion products through social media was not accessible. Though convenience sampling may constitute a generalizability issue, researchers suggested that young samples are more accurate and knowledgeable of social media and fashion products (Gautam and Sharma, 2017; Gul et al., 2021d). The reason for collecting data from youth is that they are more aware of fashion products and are more attracted to shopping online. The sample size was determined by using proposed criterion of Kline (2015). He suggested at least ten responses per item. Therefore, a minimum of 220 samples were needed, given the 22 items in this study. To increase reliability and validity, 275 questionnaires were distributed to research participants. Issock Issock et al. (2020) collected data from customers in various settings, including workplaces, supermarkets, and parks. Four Ph.D. scholars were selected as volunteers to collect data in multiple locations including shopping malls, supermarkets and universities in Shanghai the metropolitan city of China.

### Questionnaire and Measurement

Before drawing the questionnaire items, we studied and undertook a detailed literature review related to all study variables. A total of 22 items were adapted to create the final questionnaire, and these items were divided into five sections. First, remuneration motivation was measured with three items adapted from Muralidharan and Men (2015). Second, social motivation was measured with five items adapted from Wang et al. (2015). Third, empowerment motivation was measured with three items adapted from Men and Tsai (2012). Fourth, consumer commitment was measured with four items as derived by Vohra and Bhardwaj (2019). Finally, online purchase intentions were assessed with seven items adapted from Duffett (2015). All items were measured on a five-point Likert scale.

### Demographic Profile of the Respondents

The demographic analysis results showed that 53% of the respondents were male, and 47% were female; participation in both the sample assures the inclusion of genders in the dataset. About 40% of the respondents were aged between 18 and 25 years, followed by 35% aged between 26 and 35 years, and the rest of 27% were above the age of 35 years. Respondents were well-educated, with about 45% having graduation degrees, and about 49% of respondents were working in well-reputed organizations. With respect to social media type, 35% of the respondents were using Facebook, and 29% were using Instagram. About 51% of the respondents reported that they actively spend 1–3 h on social media per day.

## Data Analysis

### Statistical Model Applied

This research employs a partial least square modeling technique instead of other co-variance-based approaches such as LISREL and AMOS. The reason behind why we pick PLS-SEM is that it is most suitable for confirmatory as well as exploratory research (Hair et al., 2016). Structural equation modeling (SEM) has two approaches: covariance-based and partial least square SEM. PLS is primarily used to validate hypotheses, while covariance-based (CB)-SEM is most advantageous in hypothesis expansion. A PLS-SEM-based methodology would be done in two phases, first weighing and then measurement. PLS-SEM is ideal for a multiple-order, multi-variables model (Sarstedt et al., 2014). To do small data analysis is equally helpful in PLS-SEM. PLS-SEM allows it easy to calculate all parameter calculations (Usman Shehzad et al., 2022). The present analysis was conducted using Smart PLS 3.9.

### Model Measurement

Table 1 explains that the present study model is based on 22 items of the five variables. The reliability of this study model is measured with Cronbach’s alpha (Hair et al., 2016).

**Table 1:** Inner model evaluation.

Variables	Constructs	Factor Loading	CR	*α*	AVE
Consumer Commitment	CC1	0.778	0.834	0.733	0.557
	CC2	0.789			
	CC3	0.718			
	CC4	0.695			
Empowerment Motivation	EM1	0.741	0.853	0.770	0.593
	EM2	0.791			
	EM3	0.753			
Online Purchase Intention	OP1	0.674	0.806	0.741	0.681
	OP2	0.734			
	OP3	0.650			
	OP4	0.676			
	OP5	0.677			
	OP6	0.718			
	OP7	0.668			
Remuneration Motivation	RM1	0.773	0.821	0.773	0.605
	RM2	0.824			
	RM3	0.734			
Social Motivation	SM1	0.754	0.854	0.786	0.540
	SM2	0.688			
	SM3	0.821			
	SM4	0.731			
	SM5	0.670			

It has been shown in Table 1, all item’s reliability is robust; as it can be seen in Table 2, Cronbach’s alpha (α) is greater than 0.7. Moreover, composite reliability (CR) fluctuates from 0.80 to 0.854, which surpassed the prescribed limit of 0.70 (Chin, 1999), affirming that all loadings used for this research have shown up to satisfactory indicator reliability. Ultimately, all item loadings are over the 0.6 cutoffs which meet the threshold (Henseler et al., 2009).

**Table 2:** Mediation effects.

Relationship	Direct effect	Indirect Effect	Total Effect	VAF	Interpretation	Findings
RM → CC → OPI	0.053 (4.922)	0.073 (4.079)	0.073 (4.079)	54.07	Partial Mediation	H5a, Supported
SM → CC → OPI	0.159 (3.211)	0.064 (3.102)	0.064 (3.102)	47.87	Partial Mediation	H5b, Supported
EM → CC → OPI	0.279 (4.987)	0.133 (4.043)	0.133 (4.043)	67.34	Partial Mediation	H5c, Supported

The Cronbach’s alpha value for all constructs must be greater than 0.70 is acceptable (Hair et al., 2014). Therefore, all the values of α are greater than 0.7, as shown in Table 1; Figure 2.

**Figure 2:** Cronbach alpha.

Convergent validity is measured by CR and AVE and scale reliability for each item (Hair et al., 2016). The scholar says that CR and AVE should be greater than 0.7 and 0.5, respectively. Using composite reliability and average variance extracted scores, convergent validity was estimated (Fornell and Larcker, 1981). It is elaborated in Table 3 average variance extracted of all the indicators is greater than 0.50, and composite reliability is higher than 0.70, which is heightening an acceptable threshold of convergent validity and internal consistency. Therefore, it is stated that a value of composite reliability, i.e., not less than 0.70 is acceptable and evaluated as a good indicator’ of internal consistency (Hair et al., 2014). Moreover, average variance extracted scores of more than 0.50 demonstrate an acceptable convergent validity, as this implies a specific construct with greater than 50% variations is clarified by the required indicators (Chin, 1999; Figure 3).

**Table 3:** Hypothesis testing.

	Hypothesis	Ptah Coefficient (*t*-value)	Confidence Interval	F square	*P* Values	Decision
H1a	EM → CC	0.421 (9.312)	0.139–0.210	0.220	0.000	Supported
H1b	EM → OPI	0.279 (4.987)	0.047–0.108	0.070	0.000	Supported
H2a	SM → CC	0.201 (4.786)	0.025–0.056	0.048	0.000	Supported
H2b	SM → OPI	0.159 (3.211)	0.009–0.038	0.025	0.001	Supported
H3a	RM → CC	0.231 (4.922)	0.033–0.074	0.057	0.000	Supported
H3b	RM → OPI	0.053 (4.922)	−0.003–0.008	0.063	0.023	Supported
H4	CC → OPI	0.315 (5.097)	0.064–0.139	0.087	0.000	Supported

**Figure 3:** Measurement model.

This study determines the discriminant validity through two techniques named Fornell–Larcker criterion and heterotrait–monotrait (HTMT; Hair et al., 2016). In line with Fornell and Larcker (1981), the upper right-side diagonal values should be greater than the correlation with other variables, which is the square root of AVE, which indicates the discriminant validity of the model (Fornell and Larcker, 1981; Hair et al., 2016). Table 4 states which discriminant validity was developed top value of variable correlation with itself is highest. Furthermore, the HTMT ratios must be less than 0.85; although, values in the range of 0.90–0.95 are appropriate (Hair et al., 2016). Table 3 shows that all HTMT ratios are <0.90, reinforcing the statement that discriminant validity was supported in the present study’s classification.

**Table 4:** Discriminant validity.

Fornell–Larcker criterion						Heterotrait–monotrait (HTMT) ratios					
	CC	EM	OPI	RM	SM		CC	EM	OPI	RM	SM
CC	0.746					CC	0.669				
EM	0.681	0.762				EM	0.842	0.726			
OPI	0.633	0.618	0.686			OPI	0.832	0.672	0.814		
RM	0.625	0.626	0.528	0.778		RM	0.705	0.773	0.802	0.710	
SM	0.593	0.575	0.541	0.649	0.735	SM	0.786	0.678	0.875	0.798	0.778

CC, consumer commitment; EM, empowerment motivation; OPI, online purchase intention; RM, remuneration management; SM, social motivation.

To check the collinearity issues of the Framework, this analysis calculated the VIF values. According to the scholars, if the VIF value is less than 5, this implies no collinearity problems in the results (Hair et al., 2014; Jamil et al., 2021c). The analysis showed that the inner VIF of items falls between 1.321 and 1.876. The present study’s data demonstrate no collinearity problem with the data, and the findings are stable. An appropriate model is indicated by *R*^2^ > 0.5 in preliminary results. In Figure 2, the value of R Square greater than 0.5 on all exogenous constructs, which also means that the model has solid predictive accuracy. Q2 values of all five latent variables suggest that the model is highly predictive (Hair et al., 2016).

This study evaluates the significance of relationships by using bootstrapping at 5000 with replacement sample (Hair et al., 2016). The above table illustrate that consumer commitment has significant relationship with online purchase intention (*β* = 0.315, *t* = 5.097, *p* = 0.000). Empowerment motivation has significant relationship with consumer commitment (*β* = 0.421, *t* = 9.312, *p* = 0.000). Empowerment motivation has significant relationship with online Purchase Intention (*β* = 0.279, *t*-value = 4.987, *p* = 0.000). Remuneration motivation has significant relationship with Consumer Commitment (*β* = 0.231, *t* = 4.922, *p* = 0.000). Remuneration motivation has significant relationship with Online Purchase Intention (*β* = 0.053, *t* = 4.922, *p* = 0.023). Social motivation has significant relationship with consumer Commitment (*β* = 0.201, *t* = 4.786, *p* = 0.000). Social motivation has significant relationship with Online Purchase intention (*β* = 0.159, *t* = 3.211, *p* = 0.000). The results show that, H1a, H1b, H2a, H2b, H3a, H3b and H4 are accepted (Figure 4).

**Figure 4:** Structural model.

### Mediation Analysis

To determine the mediating role of consumer commitment between empowerment motivation, environment management, social motivation, and online purchase intention used the VAF technique (Hair et al., 2016). The value of VAF greater than 80% shows full mediation. In comparison, the value of VAF greater than 20% and less than 80% indicates partial mediation for mediation effects, and the VAF value less than 20% indicates no mediation. The results illustrate that Consumer commitment partially mediates the relationship between Empowerment motivation and Online purchase intention with direct effect. The findings show that Consumer commitment partially mediate the relationship between Empowerment motivation and online purchase intention where the direct effect (*β* = 0.279, *t* = 4.987, value of *p* = 0.000) and indirect effect (*β* = 0.073, *t* = 4.079, value of p = 0.000) with VAF 67.34% show partial mediation. The variance accounted for (VAF) describes the size of the indirect effect with the total effect. Consumer commitment partially mediate the relationship between Social motivation and online purchase intention where the direct effect (*β* = 0.159, *t* = 3.211, value of p = 0.000) and indirect effect (*β* = 0.064, *t* = 3.102, value of p = 0.000) with VAF 47.87%. Consumer commitment partially mediate the relationship between Remuneration motivation and online purchase intention where the direct effect (*β* = 0.053, *t* = 4.922, value of p = 0.000) and indirect effect (*β* = 0.073, *t* = 4.079, value of p = 0.000) with VAF 54.07%. According to Nitzl et al. (2016), a partial mediation indicated where the direct and indirect effects are significant.

## Discussion

We examined consumer motivations’ direct and indirect impact on online purchasing intentions, mediated by customer commitment within social media environments on UGT and TRA. Social media companies expend a great deal of time and effort in marketing their brands. However, there is nevertheless still interest in the online world to identify means of developing customer commitment. In this research, we emphasized that the three motives of customers, namely remuneration, socialization, and empowerment, are essential factors for developing customer commitment in marketing through social media (Yee et al., 2021).

The H1a and H1b findings revealed that remuneration motivation significantly enhances consumers’ commitment and purchase intention from online retailers. According to the present results, if consumers believe that their desires for rewards will readily be fulfilled, they are more dedicated to purchasing from asocial media platforms. Furthermore, current results show that different incentives offered from online retailers such as gifts, discounts, free home delivery, etc. are expected to produce a higher level of consumers’ commitment to online retailers, leading to higher online purchase intentions. These results comply with past study of McClure and Seock (2020), which suggest that financial and non-financial incentives affect the commitment of customers and their decision to buy online or offline, while the results contradicted the study of Cao et al. (2021).

The findings of H2a and H2b have shown the positive impact of social motivation on both customer commitment and online purchasing. It should be noted that users usually request peer reviews before purchasing products online. Results further indicate that consumers will be more committed to purchasing online before online purchasing; usually, consumers seek reviews from peers about the product and find positive reviews. This finding shows empirically what Tajurahim et al. (2020) propose and suggest that consumer will be more committed to purchasing online if he finds positive reviews from peers, but these findings earlier opposed by Lin et al. (2019). The findings also show that consumers’ intentions to purchase products online are significantly affected by the consumers’ social motivation, i.e., peer contact, which was compatible with previous research.

The H3a and H3b findings suggest that consumer commitment to purchase from online retailers is significantly and positively affected by the empowerment motivation of consumers. This finding is in line with past research, which concluded that empowerment has a significant impact on consumer commitment. However, in connection with social media marketing, this is a recent finding. This means empowering consumers by offering retailers and customers the opportunity to express their views and listen to their suggestions to better products and services, helping businesses achieve the commitment of consumers to them this finding is parallel with the prior study of Shujaat et al. (2021). Again, it is a new finding that the literature has not discussed before.

In keeping with H4, the findings indicate that customer commitment plays a significant role in purchase intentions. Furthermore, the findings show that increased commitment in online and social media marketing settings contributes to positive behavioral and attitude results. These findings are also supported by Oghazi et al. (2018) in their research. Finally, it was seen that the relationship between remuneration, social and empowerment, and online purchase intention is mediated by consumer commitment (H5a, H5b, and H5c). Thus, the relationship between consumer motivations and online purchase intentions is partially mediated by consumer commitment. These results are supported by previous studies that established consumer commitment as a significant mediating variable. Results further indicate that consumer commitment is a mediating variable that helps transmit consumer motivations toward online purchase intentions. Accordingly, consumer commitments should be placed at the forefront of evolving consumer behavior analysis models in social media settings.

## Theoretical Implications

This study provides various significant theoretical outcomes in the literature of consumer behavior. First, it enhances the understanding of consumer commitment toward online retailers and its role in developing the online purchase intentions of consumers in fashion retailing. Second, it adds to the literature on consumer commitment by concentrating on consumer motivations and desires. Researchers have shown that motivation must be seen because of its significance in consumer behavior (Rehman et al., 2019). Still, few studies exist that specifically studied the combination of different consumer motivations that influence consumer commitment toward online purchase intention. From the theoretical perspective, our study’s principal contribution is to the development and testing of the three factors of customer behavior, i.e., consumer motivation and their role toward consumers’ online purchase intention and consumer commitment to purchase fashion products online by applying UGT and TRA. These both theories provide the basis for understanding the interaction between consumer motivations, commitment toward online retailers and consumers intention to purchase online.

This study also contributes to the existing literature on consumer behavior by discussing consumer motivations (i.e., social, empowerment, remuneration) to influence consumer commitment. In this study, remuneration motivation to consider consumers’ effect on their commitment toward retailers on social media is included. Previous research focused on remuneration motivation on consumer participation with social media contributions (Irshad et al., 2020). This study contributed to the body of knowledge on customer commitment toward online purchase intentions and looked into remuneration motivation. Furthermore, the research included social motivation in this study. In the present era, social media’s primary purpose is to share views and experiences. This was the basis for using socialization motivation in the study model. Socialization is, in other words, the critical element of social media. So, by analyzing the effect of socialization motivation on customer commitment, our research adds to the literature.

Furthermore, we have included in the model empowerment motivation. Although efforts were made to define the importance of empowering the consumers while they purchase products online, this concept directly affects the consumers’ engagement behavior (Zhao et al., 2019). Therefore, all three forms of consumer motivation have shown their importance in impacting consumer commitment toward social media retailers.

*Via* the mediation path of consumer commitment in social media, the research thus enhanced the growing understanding of the effects of consumer motivations directly on intention to purchase online and mediated through consumer commitment. The significance of all hypotheses for mediation between consumer motivations and their online purchase intentions highlights that consumer commitment toward online retailers constitutes a significant mediating factor. To test the hypotheses, the data were collected from young customers in the fashion industry to understand the interplay of consumer motives toward online purchasing their commitment toward intentions to purchase online (Chen and Qasim, 2021). Most of the previous studies in online purchasing did not focus on a specific industry and specify the group of the population, i.e., young consumers. Therefore, our study provides deep knowledge and a significant contribution to online retailing digital marketing literature as its main focus is fashion products and young consumers.

## Practical Implications

The present study has significant managerial implications for retailers working on social media. Since social media marketing remains embryonically challenged in China, including consumer trust, retailers are expected to focus their marketing strategies on fostering consumer trust, leading to consumer commitment toward retailers (Imtiaz et al., 2019). Based on our study’s findings, it is recommended that online retailers adopt measures to motivate the consumers, which will enhance consumer commitment. Our research shows that social motivation is the strongest predictor to develop consumer commitment, which ultimately leads to strengthening the consumers’ intention to purchase online. Emphasized that China is a collectivist system in which the social links and contact between consumers are strongly affected. Therefore, retailers in both the offline and online worlds should also take due care of their peers. Online retailers have to keep close attention to their social media pages, and reviews from customers since these communications are likely to influence the interest of consumers and their online purchase intentions. Fashion retailers can provide a range of interactivity opportunities for members and add certain networking features important to all social media community members. They stressed that retailers’ pages on different social media sites could help decide consumers to purchase online from that particular retailer. Online retailers can also foster conversations by allowing consumers to debate the newly introduced designs of their accessories with their peers and create an awareness of affiliation by adding to their affinity in the context of other users. Positive suggestions from peers will improve customer commitment and buying intentions, as Manzoor et al. (2020) emphasized. Moreover, it can be a source of positive feedback to provide enhanced informative content about fashion products, appealing product style, and product availability. Careful scans of community interactions and social media messages can help retailers develop enhanced product designs and better approaches for customer satisfaction.

Moreover, retailers should be made aware that social media consumers want exclusive product deals and incentives that can help to fulfill their financial needs, which will lead to commitment. Chinese consumers, especially young consumers, are known as reward seekers because they admire the cash benefits provided by marketing activities (Rehman et al., 2019). Therefore, fashion retailers should also attempt to attract consumers by providing exclusive promotional offers, discounts, and free vouchers. In addition, they can update on upcoming promotions and offers on social media pages to mentally prepare for the product and be excited about it. In addition, there are several religious, traditional, and national festivals in China that raise consumers’ demand for fashion items (Irshad et al., 2020). Thus, monetary and non-monetary incentives can be very effective in boosting customers’ confidence and online purchases during these festivals. Furthermore, these rewarding techniques may make consumers feel responsive and a member of a particular fashion retailer club capable of fostering commitment and increasing their intention to purchase online.

Social media enables customers to communicate their ideas and opinions to retailers and other consumers in this digital era. In light of this fact, Chinese online retailers should be aware of this and close connection with their customers. They should regularly connect with their customers and focus on the recommendations and suggestions from them to improve product quality and design. They should promote friendly, genuine, and authentic dialogs in their social media platforms with consumers. They should make it apparent that all consumers are essential, and at their end, they would do whatever to meet their wants. Their replies to customer inquiries and complaints should be timely. Their recommendations and feedback must be highly concerned. Their opinion on social media brand pages should be open to the public. Online fashion retailers in China should recognize that building customer trust in the digital age is an absolute need and will inevitably lead to increased trust in social media and the overall intention to purchase online.

## Limitations and Future Directions

The significance of this study is twofold: it contributes to researchers investigating consumer behavior and social media marketing and to academics and practitioners involved in that field. This combination of literature works in our model will lead to new linkages and a greater understanding of current knowledge. We use evidence from China, an emerging developing economy on the globe, to assess our assertions. We recognize some limitations. First, in a specific online setting, we have tested our theoretical framework. Our results cannot thus be generalized in other contexts. We motivate scholars in different economic sectors to test our model. Secondly, the study uses the cross-sectional research design, which represents static associations among variables. Since cross-sectional data capture the relations of the variables at one point in time, it can be identified as quirks if data were captured over other intervals. Thirdly, we collected data from only three cities owing to time and budgetary restrictions. We thus welcome more investigations to duplicate and test our measurement items from other populations. Finally, future researchers should add other dimensions of consumer motivations to the model, and the moderator will further strengthen the model.

## Data Availability Statement

The raw data supporting the conclusions of this article will be made available by the authors, without undue reservation.

## Author Contributions

All authors listed have made a substantial, direct, and intellectual contribution to the work and approved it for publication.

## Funding

This work was supported by the “Does buying a marriage house for children lead to poverty: From the perspective of intergenerational transfer in rural families,” 2021 Graduate Innovation Fund of Shanghai University of Finance and Economics (CXJJ-2021-342).

## Conflict of Interest

The authors declare that the research was conducted without any commercial or financial relationships that could be construed as a potential conflict of interest.

## Publisher’s Note

All claims expressed in this article are solely those of the authors and do not necessarily represent those of their affiliated organizations, or those of the publisher, the editors and the reviewers. Any product that may be evaluated in this article, or claim that may be made by its manufacturer, is not guaranteed or endorsed by the publisher.

## Supplementary Material

The Supplementary Material for this article can be found online at: https://www.frontiersin.org/articles/10.3389/fpsyg.2022.892135/full#supplementary-material
